# Design and Analysis of Hospital Throughput Maximization Algorithm under COVID-19 Pandemic

**DOI:** 10.1155/2022/8127055

**Published:** 2022-08-11

**Authors:** Haochen Zou, Geer Jiang, Bowen Cheng, Dejian Wang

**Affiliations:** Department of Computer Science and Software Engineering, Concordia University, Montreal, QC, Canada H3G 1M8

## Abstract

Under the global pandemic of COVID-19, public health facilities, such as hospitals, are required to readjust, design, and plan a safe movement flow of people to meet the social distance rules and quarantine COVID-19 and the non-COVID-19 patients to prevent cross-infection. However, readjustments to separate patients have significantly reduced the maximum throughput of public health facilities, worsening already scarce public health resources. Therefore, this paper proposes throughput maximization algorithms based on the one-way street problem which meets the requirements of social distance rules. First, the floor plan of a hospital is transformed into a graph, each node is traversed by breadth-first search. Then, this paper considers patients' node pair sets as different set unions, the direction of edges, and the color of links based on DFS-XOR algorithm are designed to distinguish the paths of COVID-19 and non-COVID-19 patients. Finally, this paper utilizes minimum shared link algorithms to determine the minimized sharing links between paths linking different set unions and components. The throughput is maximized by reducing the number of shared links and alternating links. The results indicate that compared with the brute force algorithms, the algorithms proposed in this paper significantly improve the maximum throughput.

## 1. Introduction

The COVID-19 pandemic broke out in December 2019 and quickly swept the world, with the virus affecting the global economy and everyone's daily lives. The COVID-19 pandemic has introduced unprecedented challenges in the world. Due to the emergence and prevalence of COVID-19 and variant strains of COVID-19 such as Omicron, hospitals and other public health facilities are required to readjust, design, and plan a safe movement flow of people to meet social distancing requirements [1]. The goal is to isolate COVID-19 patients from non-COVID-19 populations to avoid crossinfection and thereby reduce the number of COVID-19 cases [2]. However, although the redesigned flow of movement meets the requirements of social distance, the ability of public health facilities to accommodate patients is significantly reduced due to the need for extra spaces. This worsens the already strained public medical resources. At the same time, doctors and nurses may also be infected with COVID-19 during work and leave their posts, which exacerbates the shortage of hospital staff and further reduces hospitals' patient intake levels [3]. Therefore, this paper intends to solve the problem of how to redesign and plan the movement routes of people in hospitals and other public health facilities under the premise of meeting the requirements of social distancing in order to maximize throughput.

The arrival of infectious variants of COVID-19, such as Omicron, has led to an exponential and dramatic increase in confirmed COVID-19 cases in a relatively short period, and the number of patients needing to visit public health facilities grows as well [4]. Much of the disaster planning in hospitals around the country addresses overcrowded emergency departments and decompressing these locations. However, in the case of COVID-19 pandemic, intensive care units, emergency departments, and medical wards ran the risk of being overwhelmed by a large influx of patients needing high-level medical care [5]. Sarier et al. contradistinguished the number of patients attending the hospital urology clinic during the first year of the COVID-19 pandemic compared to 2018 and 2019 [6]. Previous works have been conducted to modify and deploy existing hospital consultation plans to quickly care for large numbers of medically complex patients. These studies are designed to maximize the throughput of patients that hospitals can accommodate. Bowden et al. described a scale-up approach to managing residents' clinical practices during the COVID-19 pandemic. Their study provides a framework for maximizing patient admission while also leveraging a broad clinician workforce, minimizing exposure, and maximizing the pool of clinicians who may not be involved in inpatient care [5]. However, their study is aimed at describing a scale-up approach to managing residents' clinical practices during the COVID-19 pandemic, targeting physicians rather than hospitals, since the situation of physicians varies greatly from hospital to hospital. Therefore, although the plan has been successful in their institutions, it needs to be significantly modified for other public health facilities. Meanwhile, their plan does not consider the social distance rules. Shahverdi et al. proposed models for assessing strategies for improving hospital capacity for handling patients during the pandemic [7]. It enables hospitals to repurpose space, modify operations, implement crisis standards of care, collaborate with other health care facilities, or request external support, thereby increasing hospital capacity. However, the strategy evaluation model they designed is mainly focusing on the routine emergency and emergency care under the pandemic, which is difficult to apply to the overall situation of hospitals and other public health facilities. Meanwhile, only a fraction of all COVID-19 cases requires emergency care, meaning that the majority of COVID-19 patients will not benefit from the above strategic assessment model [8]. Olanipekun focuses on preventing delays in transferring patients to long-term lower acuity level nursing facilities, reducing length of hospital stay, improving patient flow, and ultimately freeing up hospital beds for incoming COVID-19 patients [9]. The above-described approach maximizes the throughput of patients. However, the process involves transferring patients to nursing facilities to shorten the length of stay, rather than improving hospitals' own situations.

Therefore, in addition to the approaches discussed above, this paper is aimed at designing hospital throughput maximization algorithms which meet the requirements of social distance and can be widely implemented by most hospitals and other public health institutions. Based on the aforesaid objectives, we first transformed the floor plan of a hospital into a strong orientation connected graph for implementing graph algorithms [10]. Then, the patient node pair sets are treated as the union of different sets, the direction of edges, and the color of links are assigned based on the DFS-XOR algorithm to distinguish the walking paths of COVID-19 and non-COVID-19 patients. Finally, the minimum shared edge algorithm is implemented to determine the minimization of shared links between paths connecting different sets of unions and components. The maximized throughput is achieved by reducing the number of shared links and alternating links. The contrast experiment indicates that compared with brute force algorithm to split the walking paths of COVID-19 and non-COVID-19 patients, the algorithm proposed in this paper improves the maximum throughput of patients in public health institutions such as hospitals.

## 2. Materials and Methods

### 2.1. Convert Hospital Floor Plans to Graphics

The throughput maximization algorithm proposed in this paper is based on the graph algorithm. Therefore, the first step of the method is to transform the floor plans of hospitals and other public health facilities into graphs. A floor pan of the McGill University Health Centre is displayed in Figure 1. The graph is composed of the set of nodes and the set of edges. Nodes can be further divided into ordinary nodes and special nodes [11]. In a hospital floor plan, the corridors are the edges of the graph.

The entrances or exits of rooms can be considered as the ordinary nodes of the graph. The main entrance of the floor, the main exit of the floor, and the intersections of the corridors are decided as the special nodes of the graph.

Based on the above definition of nodes and edges in the graph, the hospital floor plan can be transformed into an undirected graph *G* = (*V*, *E*), where *V* is the set of nodes and *E* is the set of edges. Automatic understanding of floor plan images and converting floor plans to graphs could be accomplished by the deep recognition framework proposed by Lu et al. [12]. A sample of transformation and the result are displayed in Figure 2.

Under the background of the COVID-19 pandemic, some consulting rooms of hospitals are required to treat the COVID-19 patients; the other consulting rooms are receiving non-COVID-19 patients [13]. In public health, social distancing, also called physical distancing, is a set of nonpharmaceutical interventions or measures intended to prevent the spread of a contagious disease by maintaining a physical distance between people and reducing the number of times people come into close contact with each other [14]. Canada adopted a two-meter (approximately 6 ft) social distancing policy [15]. Although the requirement of social distance in public places has been gradually abolished, the restriction of social distance is still strictly enforced in public health facilities such as hospitals [16].

Hospital corridors are clearly inadequate for social distance rules, especially when there is a large flow of people. Therefore, COVID-19 patients and other patients cannot share the same corridor at the same time. When one corridor is shared by both COVID-19 patients and other patients, we consider the edge of this corridor as the shared edge.

Therefore, the hospital floor plan further consists of the following parts: consulting rooms for COVID-19 and non-COVID-19 patients with entrances and exits, the main entrance and exit of the floor, corridors for patients to move, and intersections of corridors. The sample floor plan of a hospital in a graph with COVID-19 and non-COVID-19 node sets is displayed in Figure 3.

The hospital floor plan is eventually converted into an undirected graph. In the graph, we require that each consulting room must have (1) at least one path from the main entrance of the floor to the entrance of the consulting room; (2) at least one path from the exit of the consulting room to the main exit of the floor; and (3) at least one path from the exit of any consulting room to the entrance of any other consulting room within the same node set, to meet the accessibility. Therefore, there must be some edges that need to be considered as shared edges as defined above. In the graph algorithm, the edge is undirected, and the link is directed [17]. The flow of people on one edge can be maximized when the edge is oriented as a one-way link, while to satisfy the accessibility, some of the edges must be determined as two-way links; these links are defined as alternating links. Alternating links are the links that are used in both directions, utilized alternately in each direction, with the usage of a single direction at any given time and a waiting area at each end of the links associated with alternating links. Throughput is rate of production or the rate at which something is processed [18]. In the context of the paper, throughput is the number of people reaching their destination per time unit [19]. As the shared links defined and discussed above, the existence of alternating links and shared links reduces the throughput of patients in a hospital because when one group is passing, the other group must stay at one end and wait, which significantly weakens the traffic efficiency of the flow. Shared links and alternating links contain waiting areas at their origins, which correspond to converge flows, and therefore lead to a source of flow slowdown [20].

Hence, the essence of the throughput maximization algorithm is to minimize the number of shared links and alternating links in the graph of the hospital floor plan.

### 2.2. Label Colors of the Edges

Given the undirected graph of a floor plan *G* = (*V*, *E*) computed from the above section, two sets of node pairs are generated: SD1: the non-COVID-19 node pairs set, and SD2: the COVID-19 node pairs set. Sample SD1 and SD2 is shown in Figure 3, as the non-COVID-19 and COVID-19 patients consulting room entrances and/or exits separately. Nodes from SD1: *s*_1_, *s*_2_, ⋯, *s*_*n*_ ∈ *V*. Nodes from SD2: *s*_1_′, *s*_2_′, ⋯, *s*_*n*_′ ∈ *V*. Particularly, special nodes can be considered as belonging to both node pairs set, as the main entrance of the floor, the main exit of the floor, and the intersections of the corridors can be passed by both non-COVID-19 and COVID-19 patients. Corridors *l*_1_, *l*_2_, ⋯, *l*_*n*_ ∈ *E*. The goal is to label the same color link paths for individual node sets, such that COVID-19 patients walk along the red color link paths, and non-COVID-19 patients walk along the green color link paths, therefore, to detect all edges *l* ∈ *E* and *l*′ ∈ *E* in the graph *G* where *l*(*u*, *v*), *u* ∈ SD1, *v* ∈ SD1, and *l*′(*u*′, *v*′), *u*′ ∈ SD2, *v*′ ∈ SD2.

The breadth-first search (BFS) algorithm is implemented on the undirected graph *G* = (*V*, *E*) to make sure that all nodes in each set are reachable from the root nodes which are the main entrance [21]. The algorithm is described below in Algorithm 1.

Apply BFS search with the condition that only the node with SD1 or SD2 sets can be added to the queue [22]. The breadth-first tree formed after running the traditional algorithm may not visit all the vertices in some graphs for instance directed cyclic and acyclic graphs. Therefore, the traversing may be incomplete. We traverse the graphs with the usage of a modified BFS algorithm discussed below in Algorithm 2 [23].

The result of Algorithm 1 and Algorithm 2 will be the data structure of linked list as edges to form a path. It stores the node objects for COVID-19 patients and non-COVID-19 patients. We implement a Color Path Algorithm to color the original graph with two undirected paths consists of edges, as discussed in the Algorithm 3.

The total running time of the proposed algorithm is *O*(*V* + *E*) [24], since the most time taken part is custom BFS by using the linked list data structure to store the whole graph. After above steps, two datasets are formed. There are two undirected paths in the datasets. One is for COVID-19 patients, and the other one is for non-COVID-19 patients.

### 2.3. Define Orientation to Minimize Alternating Links

In this section, we define the orientation of edges in the undirected paths. The aim is to minimize the alternating links in the process of orientation, and meanwhile, satisfy the requirements of accessibility. The one-way street problem is a graph orientation problem, which means to define the orientation of edges (undirected links) subject to conditions [25]. The definition of the one-way street problem is as follows: consider an undirected graph, is it possible to choose a direction for each edge, turning it into a directed graph that has a path from every vertex to every other vertex [26]? Strongly connected components satisfy the requirement of the one-way street problem [27]. Therefore, we need to detect the strongly connected components inside each graph formed by the undirected paths.

For the two undirected graph generated by the two undirected paths, we first consider all the edges as alternating links to make the graph directed. Then, we detect the strongly connected components inside the graph. If inside the node sets, there exist cycle component connected nodes, the direction of the links formed the cycle can be defined as one side, and the cycle is considered as strongly connected component [28]. Otherwise, inside the component, some nodes may not be reachable under the one-direction way street problem's condition; hence, alternating links will be implemented. The direction of a strongly connected component cycle path will be defined from the entry to the exit or vice versa. The DFS-XOR algorithm is implemented for detecting whether there are cycle components in the graph or not as Algorithm 4 displayed below.

The total running time of the proposed algorithm is *O*(*V* + *E*) [29], since the most time taken part is custom depth-first search (DFS) by using the queue data structure to store the whole graph. The graph with define orientation paths after processing the cycle detection algorithm is displayed in Figure 4.

### 2.4. Define Orientation to Minimize Shared Links

We intend to confirm the orientation of the left alternating links in the graph, detect, and minimize the shared links to achieve the goal of maximum throughput. The current graph of a floor plan is shown in Figure 5. As displayed, there are links with already defined orientation, such as the red links and the green links in the graph. There also exist alternating links which required to be further oriented, such as the grey links in the graph.

A strong orientation is an orientation that results in a strongly connected graph. Robbins' theorem states that a graph has a strong orientation if and only if it is two-edge-connected, for example, if the graph has no bridge assuming the graph is connected [30]. An orientation of a graph *G* is an assignment of a direction to each edge of *G*, which obtains, as a result, a digraph. Let *G* be a connected graph and *B* be one of its edges. We define *B* as a bridge of *G* if the graph *G*1 obtained by removing *B* from *G* is disconnected [31]. We can conclude from the above description that the shared link is the bridge.

Identification of bridges can be done in linear time using Trajan's algorithm [32]. Multiple techniques can be implemented to minimize the number of shared links. Computing a Hamiltonian path or a cycle (Hamiltonian path with the option of going several times through the same nodes) is a mechanism for reducing the number of shred links [33]. The algorithm to compute a Hamiltonian path or a cycle is the DFS and backtracking algorithm [34]. Overall, the minimum shared edges (MSE) problem is defined as follows.

Given a directed graph *G* = (*V*, *E*), two special nodes *s*, *t* ∈ *V*, and integer *k* > 0. Find a set *P* of *k* paths from *s* to *t* in *G* so as to minimize *c*(*P*) = ∑_*e*∈*E*_*λ*(*e*), where *λ*(*e*) = 0 if *e* is used in at most one path of *P*, and *λ*(*e*) = 1 otherwise. An edge *e* with *λ*(*e*) = 1 is called a shared edge. As discussed by Omran et al., the MSE problem is NP-hard [35].

We implement a modified depth-first search (DFS) method to detect and minimize the number of bridges. The DFS algorithm generates four types of links: tree, forward, backward, and transversal [36]. Consider the DFS algorithm, while we are looking for vertices adjacent to vertex *v*, will be a bridge if and only if none of the vertex's *u* or any of its descendants in the DFS traversal tree has a back edge to vertex *v* or any of its ancestors. We can check the existence of back edges in *O*(*V* + *E*) time as the domain time to do the depth-first search. Let TIN(*v*) denotes the entry time for node *v*. We introduce an array LOW which will let us check the fact for each vertex *v*. LOW(*v*) is the minimum of TIN(*v*), entry times TIN(*p*) for each node p that is connected to node *v* via a back-edge (*v*, *p*), and the values of LOW(*w*) for each vertex *w* which is a direct descendant of *v* in the DFS tree:

(1) $$\begin{array}{c} \text{LOW}\left(v\right)=\left\{\begin{array}{c} \text{TIN}\left(v\right),\\ \text{TIN}\left(p\right),\text{for all p such that }\left(v,p\right)\text{ is a back edge},\\ \text{TIN}\left(v\right),\text{for all w such that }\left(v,w\right)\text{ is a tree edge}. \end{array}\right. \end{array}$$

After the above processes, there is a back edge from vertex *v* or one of its descendants to one of its ancestors if and only if vertex *v* has a child *w* for which LOW(*w*) ≤ TIN(*v*). If LOW(*w*) = TIN(*v*), the back edge comes directly to *v*; otherwise, it comes to one of the ancestors of *v*. Therefore, the current edge (*v*, *w*) in the DFS tree is a bridge if and only if LOW(*w*) > TIN(*v*) [37].

The minimized number of shared links is detected according to the method. The shared link is used by both COVID-19 and non-COVID-19 patients; therefore, such should be orientated in both directions.  Figure 6 shows the graph of a hospital's floor plan with the designed movement flow of patients after all the algorithms' modifications. In the movement flow designed in the figure, the maximum throughput of the floor plan is obtained by reducing the number of alternating links and shared links.

## 3. Results and Discussion

### 3.1. Results

This section presents the analysis result of the designed hospital throughput maximization algorithm. There are two crowd movement path flows for one general hospital; one is according to the brute force method, and the other one is designed based on maximum throughput algorithm proposed in this paper. We establish the crowd flow simulation model of two different paths to calculate and count the time of the crowd consumed by moving from the exits of the consulting rooms to the main exit of the floor. The time difference between the two paths is compared to achieve the purpose of contradistinguishing throughput. Since throughput is the number of people reaching their destination per time unit. Based on the same amount of people in the crowd, the longer the consumption on the path, the smaller the corresponding throughput.

Pathfinder is selected for simulation in this paper. Pathfinder is a simulator based on human movement simulation. It provides users with a graphical user interface for simulation design and operation, as well as 2D and 3D visualization tools for analysing results [38]. Pathfinder utilizes a geometric model that supports 3D. This model includes rooms, doors, stairs, exits, and other structures. The three-dimensional structure diagram of a general hospital is shown in Figure 7.

The human is the main body of the simulation function, and the simulation model of the software allows to test the speed of the human, the width of the human model, the priority level, and special behaviours of the human. Pathfinder supports both steering and SFPE mobile simulation modes [39]. By using the hypothesis group in the SPFE handbook, the simulated personnel will not try to avoid each other when moving and will be crowded with each other [40]. The traveling speed of the crowd is affected by the space density of the room, and the pedestrian flow at the exit is determined by the width of the door. In the steering mode, a reasonable distance will be maintained between people [41]. If the distance between moving people and the path of the nearest point reach or exceed a certain threshold, the system will automatically select other feasible paths and change the walking path of simulated personnel. Since the steering mode is closer to the real moving situation, the paper implements the steering mode in the simulation.

In the analysis of this paper, the population in the building is divided into eight types: adult male, sick male, adult female, sick female, normal old people, sick old people, normal children, and sick children. Simulated speed and simulated shoulder width of all kinds of personnel are adjusted according to the set parameters. The average shoulder width of personnel is set as 45 cm. According to the information provided by the hospital and field investigation, during the peak period of medical treatment, the flow of people on each floor of a hospital at a certain point is about 200 people. The building area of each floor is 1,500 square meters, and the crowd density is less than one person per square meter.

The movement speed and agility of eight different categories of personnel are different [42]. In the simulation analysis of personnel flow, the proportion and speed of personnel in the simulation software are shown in Table 1.

After generating corresponding simulators from various personnel data, we input the corresponding number of simulators into the system according to the expected personnel distribution and obtain the graph of generating simulators, as shown in Figure 8.

The two kinds of hospital personnel movement paths are generated based on the brute force method and the algorithm proposed in this paper. The simulation model with simulators in consulting rooms and corridors of the hospital moving to the main exit of the floor along the movement paths is displayed in Figure 9.

In this paper, the first floor, second floor, and third floor plans of the hospital are selected for the establishment and research of simulation model. The path diagram of personnel movement is shown in Figure 10. Randomly distributed people at each floor will choose the nearest path to the exit.

The thermal map of personnel density is shown in Figure 11.

From the simulated personnel movement path and personnel density heat map, it can be seen that the randomly distributed people on the first, second, and third floors of the hospital will choose the path to the main exit of the whole floor nearby for movement. According to the statistical time, there are 450 people on the whole three floors. The total time to reach the main exit of each floor using the movement path generated by the brute force method is 335.9 seconds, while the total time to reach the main exit of each floor using the movement path generated by the algorithm proposed in this paper is 227.6 seconds. The algorithm introduced in this paper can improve the hospital throughput.

### 3.2. Discussion

The present study developed algorithms for maximizing the patients' throughput in public health institutions such as hospitals under the requirements of social distancing. Different various methods previously designed by other scholars to improve patient acceptance are the scale-up approach to managing residents' clinical practices during the COVID-19 pandemic [5], the model for evaluating strategies to improve hospital patient handling capacity during the COVID-19 pandemic [6], and the approach of transferring patients to nursing institutions during the COVID-19 pandemic to shorten hospital stay and maximize the number of patients accepted by hospitals [8]. This paper focuses on the walking path of patients in the hospital, by applying the concept of maximum flow in the field of computer science and algorithm and reducing the number of shared links and alternating links, to achieve the goal of maximization the hospital throughput. The results of comparative experiments indicate that compared with the paths generated by the brute force method, the paths designed by the algorithm proposed in this paper can improve the throughput of hospitals by nearly 1.5 times. The study extends the current literature. Researchers can expand this study by including other public health institutions and exploring other factors affecting the maximum throughput.

The maximum flow problem is a combinatorial optimization problem, which discusses how to make full use of the capacity of the equipment to maximize the flow and achieve the best effect [43]. The labelling algorithm for maximum flow was first proposed by Ford and Fulkerson in 1956. The “network flow theory” established by Ford and Fulkerson in the 1950s is an important component of network applications [44]. Network flow is a kind of specific flow solving method, which is closely related to linear programming. The theory and application of network flow are developing continuously, and new topics such as flow with gain, multiterminal flow, multicommodity flow, and the decomposition and synthesis of network flow appear [45]. Network flow has been widely used in communication, transportation, power, engineering planning, task assignment, equipment updating, and computer-aided design. In this paper, the application of the maximum flow problem is extended to medical fields such as public health facilities to meet social distancing requirements under the COVID-19 pandemic.

The COVID-19 pandemic and the emergence of COVID-19 variants such as Omicron have put a strain on already stretched public health resources, with existing facilities overwhelmed by the soaring number of people needing to visit hospitals. Based on the concept of the maximum flow algorithm, walking path algorithms satisfying social distance are designed in this paper. On the basis of the existing public health resources, the hospital can maximize the throughput of people by minimizing unnecessary waiting time and preventing dangerous situations happen such as crossinfection. At the same time, the results of this paper can also be applied to other places to prevent crossinfection of infectious diseases, such as mobile cabin hospitals. Efforts should be made to reduce the waste of public medical resources which are already scarce.

Our study focuses on developing pseudocode-based algorithms for maximizing the throughput in hospitals. Since different public health institutions implement different programming languages for their Hospital Information Systems (HIS), the original intention of designing algorithms utilizing pseudocode is to hope that public health institutions such as hospitals and clinics can implement the algorithm by themselves by applying the programming language they utilize. However, this may prove difficult. Meanwhile, when applying the algorithms to some relatively complex floor plan scenes, the results generated in each step of the algorithms may need to be slightly improved according to the actual situation. These improvements require algorithms, graph theory, and other related knowledge for relevant medical staff, which might cause inconvenience. The above-mentioned points lead to the limitations of the research. Thus, future studies should design programs and systems which can be run on portable devices [46], in order to achieve the automatic generation of walking paths that can help hospitals and other public health facilities obtain maximum flow. What is more, it is the goal of future research and works to improve the matching degree and accuracy of the results of the designed algorithm with the real public health institutions environment, so as to reduce the subsequent modification operations for medical staff. Meanwhile, future work will focus on reducing the number of iterations in the algorithm, such as loops and recursion, to improve the efficiency of the algorithm as much as possible and reduce the time and space complexity of the algorithm.

## 4. Conclusions

Due to the COVID-19 pandemic, hospitals and other public health facilities are being requested to redesign the way people walk in corridors to meet social distancing requirements. In this paper, algorithms based on the maximum flow problem are proposed in order to present movement flows and satisfy social distancing requirements. The core idea of the algorithm is to minimize the number of shared links and alternating links. The experimental results indicate that compared with the traditional methods, the designed algorithms can improve the throughput of public health institutions and achieve the aim of maximizing the usage of public medical resources.

## Figures and Tables

**Figure 1:** The floor plan of McGill University Health Centre.

**Figure 2:** A sample of transformation from a floor plan to a graph: (a) the floor plan; (b) the transformed graph.

**Figure 3:** The sample floor plan of a hospital with COVID-19 and non-COVID-19 node sets.

**Figure 4:** The graph with direction after algorithm modification.

**Figure 5:** The current graph of a floor plan with oriented links and links to be oriented.

**Figure 6:** The movement flow of a floor plan graph after algorithm modification.

**Figure 7:** The three-dimensional structure diagram of a general hospital.

**Figure 8:** The three-dimensional structure diagram of a general hospital with simulators.

**Figure 9:** The simulation model with simulators.

**Figure 10:** The path diagram of personnel movement.

**Figure 11:** The path diagram of personnel movement.

**Algorithm 1:** Breadth-first search algorithm.

**Algorithm 2:** Modified BFS algorithm.

**Algorithm 3:** Color path algorithm.

**Algorithm 4:** DFS cycle count XOR algorithm.

**Table 1:** Proportion of eight types of people and the walking speed.

Type of people	Proportion (%)	Walking speed (m/s)
Adult male	13	1.3
Sick male	25	1.0
Adult female	12	1.1
Sick female	25	0.85
Normal old people	3.25	0.8
Sick ole people	9.75	0.65
Normal children	3	1.0
Sick children	9	0.8

## Data Availability

The data underlying the results presented in the study are available within the manuscript.
